# The Role of Mastering Musical Instrument Playing Skills Combined with Student Behavior Data Mining and Analysis in the Digital Campus Environment to Improve Students' Comprehensive Quality

This article has been retracted.

**DOI:** 10.1155/2022/7724675

**Published:** 2022-09-10

**Authors:** Mengyu Shi

**Affiliations:** Music Education Theory Teaching and Research, Belarusian State Pedagogical University Named after Maxim Tank, Minsk 220013, Belarus

## Abstract

Music is closely related to people's lives, and it has a certain impact on people's lives. In school teaching activities, mastering the skills of playing musical instruments can effectively improve students' music appreciation ability and level and enhance students' comprehensive quality through subtle influence. Based on the analysis of students' behavior data, this paper analyzes the role of mastering musical instrument playing skills in improving students' comprehensive quality and puts forward research ideas and schemes. It focuses on students' group behavior in the digital campus environment, integrates multisource data in the digital campus, quantificationally calculates students' multidimensional behaviors, studies the behavior rules of students with different academic performance levels, and uses machine learning algorithm to build a multifeature integrated model of students' comprehensive quality, providing personalized feedback for the improvement of students' comprehensive quality. The results show that the effect of mastering musical instrument playing skills combined with data mining analysis of students' behavior is generally 30% higher than that of the previous research. Compared with a single model, the fused model can fully consider each algorithm to observe data from different data spaces and structures and give full play to the advantages of different algorithms. The training of a single model will fall into the local minimum, which may lead to the relatively poor generalization performance of its model. However, the weighted fusion of multiple basic learners can effectively reduce the probability of falling into the local minimum.

## 1. Introduction

Combined with the analysis of students' behavior data mining, the role of mastering musical instrument playing skills in improving students' comprehensive quality refers to the internal and relatively stable main characteristics and qualities that are formed or developed in the learning and practice of students in the education stage and have positive significance for students' sustainable development [1]. The higher the comprehensive quality, the stronger the ability of young students to understand and transform the objective world. Young students are in the golden period of life development. At this stage, they not only need to learn rich cultural knowledge and professional skills but also need to cultivate and develop their comprehensive quality [2]. This is not only the objective need of personal growth and success but also the inevitable requirement of China's economic and social development for outstanding talents in the new era. However, for a long time, influenced by various subjective and objective factors, there is still a problem of ignoring comprehensive quality education in school education in China. Even though some schools have also carried out comprehensive quality education, it is more superficial, and its educational effect is not ideal [3]. The lack of comprehensive quality education for young students easily leads to a series of problems in their learning attitude, learning ability, political literacy, moral quality, values, and so on, which greatly restricts the healthy development of young students. For young students, comprehensive quality education is an important way to cultivate their personality and develop their various abilities [4]. Young students occupy a fundamental and strategic position in the construction of socialism with Chinese characteristics. The improvement and development of their comprehensive quality are the only way to strengthen and revitalize the country. School educators should be based on the new era and fully understand the urgency and necessity of comprehensive quality education for young students from the height of national strategy [5].

Musical instrument playing covers all aspects of life, which expands and extends the value and significance of mastering musical instrument playing skills. In the process of musical instrument playing, students gain not only music knowledge and enjoyment of music art but also knowledge of history, humanities, customs, geography, and other aspects contained in playing music. For example, the invention, spread, evolution, and modern development of musical instruments are all part of musical instrument knowledge. Many classical musical instruments are artistic interpretations of historical events. Feeling historical events from music appreciation can help students better interpret historical events [6]. All over the world, the music of every nation has its unique musical instrument playing expression, which is also the concentrated expression of local customs and national customs. Students can feel the local customs and customs of all over the world by learning musical instruments. In a word, the process of mastering musical instrument playing skills contains rich elements of cultural knowledge, which can promote the improvement of students' comprehensive quality. This paper focuses on students' group behavior in the digital campus environment, aiming at integrating multisource data of digital campus, quantitatively calculating students' multidimensional behavior, studying the behavior rules of students with different academic performance levels, and using machine learning algorithm to build a model of students' comprehensive quality with multifeature fusion, so as to provide personalized feedback for the improvement of students' comprehensive learning quality. Practice has proved that combining students' behavior data has profound significance and function in exploring whether mastering musical instrument playing skills can improve students' comprehensive quality.

The coefficient of the weight of students' comprehensive quality evaluation index is the basic information reflecting the quality of students' comprehensive quality [7]. It reflects the evaluators' judgment on the importance of each index. Among all kinds of index evaluation methods, index data and index weight are the two major factors that directly affect the final result of evaluation [8]. The evaluation of students' comprehensive quality is no exception, so whether the weight coefficient of students' comprehensive quality index is designed scientifically will directly affect the scientificity and rationality of the evaluation results of students' comprehensive quality. Based on the prediction and research of students' behavior analysis, this paper adopts the computer method of pairing and sorting to predict students' behavior. Compared with the traditional prediction of students' comprehensive quality or GPA, this method pays more attention to students' individual performance and changing trend in a whole group.

This method can help the education work to continuously observe and intervene students' academic performance in the actual education and teaching work, and at the same time, it can better grasp the characteristics of different groups of students, so as to optimize the behavior research of students of different majors. Its innovation lies in the following: (1) drawing an objective and thorough “student portrait” can help students develop their self-awareness and provide direction for their self-development while also enhancing the school's capacity to recognise students' learning growth and daily behavior based on the analysis of the behavior characteristics of their personal big data. (2) Based on the analysis of students' group behavior characteristics, explore the role of mastering musical instrument playing skills in improving students' comprehensive quality. (3) Based on students' behavior data, the essential personality characteristics of students are extracted from the perspective of Big Five personality traits, and the network system of students' comprehensive quality evaluation is clearly modeled.

## 2. Related Work

After extensive accumulation and strong support from the Ministry of Education, research into educational data mining technology in China is now at a relatively advanced stage. The related research in depth and breadth of educational data mining technology is very advantageous. In order to promote the research and application of data mining technology in the field of education, it focuses not only on the improvement and optimization of data mining algorithms but also on the development of numerous mature application systems. This work has produced promising theoretical and practical outcomes.

Lu put forward an association rule algorithm and conducted data mining on the participation patterns of musical instruments [9]. Wang et al. put forward the classification algorithm and also invented a large number of relatively mature data mining software [10]. Peng put forward a new model of blended learning and introduced its learning process and learning environment [11]. Wang et al. used educational data mining methods to identify the students' situation and participation patterns in distance learning [12]. Lust et al., considering the generality of personality and group students, put forward a collaborative filtering recommendation method for students' mastery of knowledge points by using cognitive diagnosis technology [13]. Brooks has achieved satisfactory results by mining educational data and analyzing the performance of feature selection algorithm [14]. Shanabrook et al. analyzed the data of students' consumption and used data mining and statistical analysis to find out the hidden law of students' consumption behavior [15]. Rusby et al. used data mining technology to analyze students' consumption and borrowing behaviors and built a system model of students' behavior analysis. By inputting various behavior characteristics into the model, they judged whether the student's learning mode was reasonable, and the analysis results helped students find their own effective learning methods [16]. Gu and Huang, by analyzing the data of students' campus card, measured students' campus life behavior by using entropy-based measurement and reached the conclusion that there is a great correlation between the regularity of campus life and comprehensive academic achievement [17]. Zhu et al. can learn about students' learning, consumption, and work and rest behaviors through deep and systematic research on students' consumption behaviors and give early warning tips for abnormal situations [18].

The computer method of pairing sorting used in this paper can find frequent transaction item sets from massive data, so as to infer the correlation between transactions. Association rules first discussed the association of supermarket shopping baskets. Since then, many scientific researchers have also begun to be interested in association rules. The research on the theory and application of association rules has become more and more in-depth, and many improved algorithms on association rules have been published [19]. The most classic algorithms are a priori algorithm and FPT growth algorithm, but these two algorithms need to scan the database many times to produce frequent patterns and will also produce a large number of frequent item sets. Therefore, the time and space complexities are relatively large, and the operation efficiency may be low in the process of data mining. However, Eclat algorithm adopts vertical data representation, and it can quickly calculate the support of item sets by scanning data records only once, so as to improve the excavation quality.

## 3. Methodology

### 3.1. Behavior Regularity

Behavior regularity is another very important feature of the sense of responsibility in the Big Five personality, which represents students' ability of self-discipline. Compared with students with chaotic life rhythm, students with strong self-discipline usually have strong willpower and the ability to control their own lives and can properly arrange their own life and study. Such personality characteristics can positively affect students' comprehensive quality performance, so behavioral regularity is the personality characteristics that this study focuses on and discusses. This paper will study the quantitative method of behavior regularity from two parts: behavior change and behavior complexity, that is, quantify the regularity of students' behavior from linear and nonlinear angles. The quantization process is shown in Figure 1.

People with a strong sense of responsibility usually have a high ambition, pursuit, and a strong self-driving force to strive for goals. The superposition of these factors usually leads to a higher comprehensive achievement. The internal reason is that input and output are usually in direct proportion, and spending more time and energy on synthesis will usually bring better comprehensive results [20]. However, the comprehensive quality here is an abstract concept, which is not convenient for direct evaluation in teaching. How to quantify or project the comprehensive quality value to the detailed behavior of students is a problem that needs to be discussed. We need to dig deep into the time series data of students' behaviors extracted from the original one-card and WIFI data and evaluate the comprehensive quality of students according to the corresponding index characteristics. The magnitude process is shown in Figure 2.

Comprehensive quality behaviors mainly include library access control, borrowing books, and time series data of WIFI staying in comprehensive areas. The frequency of comprehensive behaviors can be directly counted to define students' diligence [21]. Frequency, that is, the number of times behavior occurs in a period of time, is a common statistical indicator. The higher the frequency, the more frequent the students' comprehensive behaviors occur in a fixed time, which is the most direct index quantification method of comprehensive diligence. For WIFI time series data, we can separately count the network connection frequency of students in different areas. From the processed data, we can observe that the most important activity places of students are the comprehensive area and the rest area, and these two areas can best reflect students' comprehensive behavior. Specifically, the online data in the comprehensive area can directly reflect the students' comprehensive state, while the online data in the rest area is the supplementary data reflecting their comprehensive behavior. This is because compared with the comprehensive area, students use the internet more frequently when relaxing in the rest area, so the amount of data in this part is far greater than that in the comprehensive area, and the time spent in the rest area is usually inversely proportional to students' diligence, which can be used to quantify this indicator in reverse.

### 3.2. Behavioral Complexity

The loose and free campus environment makes students' behavior random and diverse. In this case, the simple mathematical statistics method cannot fully study its behavioral complexity, and more effective quantitative indicators need to be discovered and used. Information entropy can effectively measure the orderly behavior of students. The calculation formula of information entropy is as follows:

(1) $$\begin{array}{c} \text{Entropy}=-\overset{n}{\underset{i=1}{\sum }}pi\log pi, \end{array}$$

where *n* is the total number of different characters in the data and *i* is a single character. Information entropy, the most fundamental index for measuring information uncertainty, can be used to quantify information uncertainty in informatics. Information entropy, however, has a significant flaw in assessing the complexity of behavior. We can determine that formula (1)'s information entropy calculation method ignores the relationship between elements and instead concentrates on the frequency of occurrence of a single element. That is to say, even if the data's internal components change, the results obtained before and after the change will be the same as long as the structure does not change.

The regularity and complexity of data in nonlinear time series are frequently examined using approximate entropy. The probability of new data patterns appearing in time series is reflected by approximate entropy, which can be used to detect data changes in complex systems. The complexity of time increases with approximate entropy. The entropy is calculated roughly as follows:

(2) $$\begin{array}{c} \text{ApEn}=\ln\overset{N-m+1}{\underset{i=1}{\sum }}C_{i}^{m}-\ln\overset{N-m}{\underset{i=1}{\sum }}C_{i}^{m+1}. \end{array}$$

∑_*i*=1_^*N*−m+1^  is the average similarity rate of all subsegments with a period of *m*, while the second half is the average similarity rate of all subsegments with a period of *m* + 1. The approximate entropy formula allows us to know that this index represents the likelihood that new patterns will appear in time series when the dimension changes. This technique is useful for assessing the structural complexity of time series.

Log refers to the debugging information of users after they connect to the campus network, in which each data line contains different response information, and different response information is also distinguished by code segments. Therefore, it is necessary to analyze the corresponding information of different codes in order to process the log data accurately. Due to the huge amount of WIFI data, there are a lot of redundant data which are repeated and not needed, so it is a complicated project to extract the required space-time information from this data. The server captures WIFI data once, counts students' online information at 1-minute intervals, divides the area by the functions of buildings on campus, and replaces the physical location of the AP end with functional areas such as study areas and rest areas. The processed space-time data is shown in Table 1.

This study obtained a large number of behavior characteristics after quantifying the characteristics of the behavior data. The correlation between two variables is measured using the correlation coefficient. Its value ranges from -1 to 1, and a positive value denotes a positive correlation between the two variables. The stronger the correlation, the larger the absolute value of the correlation coefficient. The following is the calculation formula:

(3) $$\begin{array}{c} r=\frac{\sum_{i=1}^{n}\left(xi-x\right)\left(yi-y\right)}{\sqrt{\sum_{i=1}^{n}{\left(xi-x\right)}^{2}}}. \end{array}$$

Confidence *r* is the premise used when discussing the correlation between two variables, and the absolute value of the correlation coefficient represents various correlations. If the value of *r* is too small, the calculated correlation coefficient result is not credible. In the correlation analysis of this study, when the confidence *r* value is less than 0.09, the correlation result is reliable.

GBDT algorithm uses Boosting-based ensemble learning method to iterate weak learners to form strong learners. The decision tree model of weak learners is regression tree or classification tree. The specific algorithm flow of GBDT classification algorithm is as follows.

First, initialize the weak learner, as shown in the following formula:

(4) $$\begin{array}{c} f\left(x\right)=\arg\min\overset{n}{\underset{i=1}{\sum }}L\left(yi,c\right). \end{array}$$

Secondly, the number of iterations is *s* = 1, 2, ⋯, *S*, and the negative gradient for each sample is calculated as shown in the following formula:

(5) $$\begin{array}{c} mi=\left[\frac{\partial L\left(yif\left(x\right)\right)}{\partial f\left(x\right)}\right]. \end{array}$$

Then, the residual (negative gradient) of these *n* samples is fitted by using regression tree as shown in the following formula:

(6) $$\begin{array}{c} c=\arg\min\underset{x\in M}{\sum }L\left(yi,fi-1+c\right). \end{array}$$

Finally, the strong learner is continuously updated according to formula (6), and the following formula is obtained:

(7) $$\begin{array}{c} f\left(x\right)=fs-1\left(x\right)+\overset{J}{\underset{j=1}{\sum }}cI. \end{array}$$

The final strong learner is shown in the following formula:

(8) $$\begin{array}{c} f\left(x\right)=\overset{S}{\underset{x=1}{\sum }}\overset{J}{\underset{j=1}{\sum }}cI. \end{array}$$

The formula can flexibly handle various types of data and adjust parameters in a short time and has high prediction accuracy. The loss function is used to enhance the robustness of outliers, and the weight of each classifier is considered comprehensively.

This function shows a stable advantage in quantifying behavior complexity. It uses the characteristic of the simplest and most common data change in the quantitative relationship to quantify the contingency and complexity of the behavior pattern structure. This function is similar to the calculation idea of approximate entropy, which judges the similarity between subsequences. However, the judgment methods are quite different, and the calculation dimension of this function is more diversified than that of approximate entropy. Among them, the calculation rule of *xi* is shown in formulas (9) and (10):

(9) $$\begin{array}{c} xi=\overset{L}{\underset{j=2}{\sum }}\frac{Pj}{L+j-1}, \end{array}$$

(10) $$\begin{array}{c} yi=\overset{k}{\underset{k=1}{\sum }}fk\left(xi\right), \end{array}$$

where *pj* is the change number when the time interval is *j* and the final complexity is the average value of the change number of subsequences. *pj* is calculated as follows: when *j* = 2, if the two characters are different, it will be recorded as a change, and *p* is the sum of all the changes. When *j* ≥ 2, compare whether the string formed by the first *j* − 1 and the last *j* − 1 symbols in a subsection has the same number of changes. If the number of changes is different, record it as a change, and *pj* is the sum of the number of changes of all subsections with a length of *j*. This index integrates and quantifies the structural information of time series.

According to the formula of entropy, the greater the entropy, the lower the predictability and the worse the stability of behavior. Generally speaking, students with excellent comprehensive scores have better behavior stability. In other words, there should be a negative correlation between entropy and students' comprehensive scores. However, according to the correlation coefficient results in the previous section, we can know that there is a positive correlation between entropy and students' comprehensive scores in the data set of this paper. This phenomenon is caused by the behavior characteristics of students in different comprehensive grades. Thus, the probability density function images of students' approximate entropy comprehensive indicators in different comprehensive score intervals are drawn, as shown in Figures 3 and 4.

Figures 3 and 4 depict the probability density distribution of FSA determined by various behaviors, respectively, and Figure 5 depicts the probability density distribution of FSA determined by the approximative entropy of various behaviors. The probability near a specific value of the *X*-axis is indicated by the value of the *Y*-axis in the image, and the probability in a specific interval of the *X*-axis is the integral of the probability density curve in this region.

## 4. Experimental Results and Analysis

Three models are built in the same experimental setting: a single random forest model, a GBDT model, and an Xgboost model. This is done to demonstrate the efficacy of the integrated comprehensive performance prediction model proposed in this paper. Compare the accuracy, precision, recall, and *F*-measure model evaluation indexes. The comparison results are displayed in Table 2.

As can be seen from Table 2, from the above four evaluation indexes, the three single models are generally consistent in the prediction model indexes, and the accuracy of each single model is 55.34% higher than the experimental baseline. For the random forest model, the lower the correlation of features, the better the classification effect of the model, the lower the sensitivity of the random forest to missing data, and the better the classification effect with less data, which is why the random forest model has better classification effect in the test set. For GBDT and Xgboost models, the algorithm training needs to go through many iterations, and the calculation amount is much higher than that of the random forest algorithm. By increasing the calculation complexity, the prediction performance of the model can be improved. Generally speaking, by comparing and analyzing the prediction results of students' comprehensive scores by the above three models, the Xgboost model has stronger learning ability than the characteristics of students' behaviors extracted by the random forest and GBDT model, and the accuracy and precision of the prediction model obtained by training are relatively higher, so the reliability of prediction is also relatively higher. The fusion comprehensive performance prediction model proposed in this paper is compared with the single prediction model, and the comparison results are shown in Figure 5.

In comparison to the single random forest, GBDT, and Xgboost model, the fusion prediction model proposed in this paper has significantly improved in four indexes, and its prediction accuracy is higher, making it more suitable for prediction, as shown in Figure 5, comprehensive student grades. At the same time, it is evident that a single model's classification accuracy for predicting students' overall performance is low, and algorithm optimization can only slightly enhance the accuracy of the final prediction. The choice of data features and the integration of models are what ultimately determine the model's accuracy. The rationale for why the fusion model is superior to a single model is examined theoretically. The fusion model based on the Boosting algorithm combines several classification models, allowing it to fully take into account each algorithm when observing data from various data spaces and structures and to fully exploit the benefits of various algorithms. A single model training will run the risk of a local minimum from the perspective of model optimization, which could result in a relatively subpar generalization performance. However, after weighted fusion, the likelihood of entering a local minimum can be significantly decreased by training multiple basic learners.

To sum up, the fusion of models can only improve the final experimental results to a certain extent and count the data sets. Whether the preprocessing is good or bad or whether the effective behavior characteristics that affect the comprehensive academic performance and are not extracted will affect the final result of the model is not reflected. At the same time, according to the basic principles of different algorithms, different classification models will have obvious differences in the learning of students' behavior characteristics. The extraction of students' behavior characteristics is a relatively subjective process, and the extraction of behavior characteristics that effectively affect students' comprehensive performance is not comprehensive enough, which also reflects the importance of preprocessing and data analysis.

In general, the research presented in this paper shows that it is possible to predict students' overall performance using information about their behavior. The prediction effect is constantly improving, from single prediction models to fusion models, but the actual effect of the model is not optimal overall. Analyzing the causes may reveal that the model cannot automatically learn the information from the original data and that manual statistical behavior characteristics perform poorly when applied to traditional methods. This underlines the significance of feature extraction and data analysis and indicates a path for further enhancing the accuracy of comprehensive performance prediction.

In addition, 70% of the student behavior data are chosen as training data and 30% as test data due to the sparseness of the data. The experiment makes use of the stacking feature and the CNN model as the base classifier. Numerous prediction indicators are used to gauge the effectiveness of the comprehensive performance prediction model. The CNN-LSTM network model with time series features outperforms the single CNN model when subjected to a consistent experimental environment and a set of evaluation criteria. In terms of thorough performance prediction, the CNN-LSTM network model with attention mechanism performs the best. The corresponding relationship between training times, accuracy, and loss on the test set and training set is depicted in Figures 6 and 7 below, respectively.

According to Figure 6, the model accuracy rate rises as training times increase in the training set and falls as training times rise in the testing set. It is known that the model with 12 training rounds produces the best results.  Figure 7 illustrates how, during the initial training phase, the model's loss value decreases as the number of training sessions increases and is lower during training than during testing. The analysis above demonstrates the model's strong training and testing effect.

## 5. Conclusion and Prospect

Comprehensive quality is a comprehensive cognitive ability composed of attention, observation, memory, imagination, and thinking ability. Comprehensive quality factor is an important psychological factor that marks people's quality. The human brain is a unified whole, which contains great learning and creative potential. The number of human brain cells is about 18 billion, but only more than one billion of them are always in an active state, and more than 90% of them are in a relatively static or sleeping state. In a person's life, only about 10% of brain cells are used. It can be seen that the human brain has great potential to be tapped. The ability stored in the brain makes us dumbfounded. If we can force our brains to reach half of their working capacity, we can easily learn more than 70 languages, memorize an encyclopedia of the former Soviet Union, and finish courses in 20 universities. Therefore, the right brain not only has a large memory capacity but also has incomparable advantages over the left brain in terms of cognition, such as specific thinking ability, ability to recognize space, ability to understand complex relationships, and emotional expression and recognition ability, which is superior to the left brain. Therefore, the development of the right brain function is crucial to human development. However, the traditional educational methods lay particular stress on reading, writing, mathematical operations, and rational thinking and mostly focused on the activities of the left brain, thus resulting in the overload of the left brain, while the right brain was left idle, which resulted in the incomplete development of comprehensive quality. Therefore, the revelation of brain function by brain science is of great significance to our scientific construction of quality education system. Only when the two hemispheres of the brain cooperate with each other and develop in a balanced way can people's comprehensive quality be highly developed. However, the function of the right brain is closely related to the performance of musical instruments. When playing the piano, the left and right hands alternately coordinate with each other, which promotes the coordinated development of the two hemispheres of the brain and makes the thinking more agile. Therefore, there is a scientific basis for saying that mastering the playing skills of a musical instrument is conducive to the development of comprehensive quality factors. When students play the accordion, they should simultaneously reflect the high and low spectrum tables, quickly identify the high, low, long, short, continuous, broken, strong, and weak sounds on the spectrum tables; change the speed and timbre; and control the bellows operation. Students should complete these comprehensive actions in an orderly manner at the same time and turn the music score into a vivid sound, which will undoubtedly promote the development of students' comprehensive quality factors.

Big data and artificial intelligence advancements have facilitated the digital and thoughtful transformation of conventional campus settings. In order to determine whether learning to play a musical instrument can enhance students' overall quality, this paper will analyze students' behavior using student data collected from the campus environment. The primary work contains the following:

1. In this paper, the sources and characteristics of students' behavior analysis and comprehensive performance prediction are introduced. Current data on students' behavior analysis and comprehensive performance prediction are also explained, and the methods for comprehensive performance prediction based on conventional machine learning are categorised and summarised. This paper introduces the related research and applications of deep learning and sequence modelling by analyzing the issues encountered in the construction of students' comprehensive performance prediction model
2. A data mining algorithm-based fusion model for performance prediction is created. A fusion model based on random forest, GBDT, and Xgboost is established in accordance with the conventionally manually extracted behavior characteristics. First, the weights of the single classification models for random forest, GBDT, and Xgboost are calculated using the Boosting algorithm. Next, the above single models are fused using the weighted average method. Finally, the fused model is compared to the single model to assess its efficacy

The findings demonstrate that it is possible to predict students' performance using information about their behavior. The prediction model based on attention mechanism has higher prediction accuracy and better performance compared to the prediction model based on data mining, which confirms the importance of mastering musical instrument playing skills combined with data mining analysis of students' behavior in enhancing students' overall quality. Although this paper has made some achievements in extracting students' behavior characteristics and predicting accuracy of students' grades, in the data preprocessing stage, we should study the data deeply, choose a better data cleaning method, effectively clear the abnormal data, fill in the missing data, and then do in-depth analysis of various behavior data to improve the granularity of data to find more effective behavior characteristics. Further research is needed by using the methods and ideas proposed in this paper.

## Figures and Tables

**Figure 1:** Quantification process of behavior regularity.

**Figure 2:** Quantification process of comprehensive quality value.

**Figure 3:** Probability density distribution.

**Figure 4:** Distribution of approximate entropy probability density.

**Figure 5:** Performance comparison of classification prediction models.

**Figure 6:** Accuracy curves of the test set and training set.

**Figure 7:** Loss curve of the test set and training set.

**Table 1:** Data table of students' time and space after processing.

Student number	Time	Location	Capture times	SNR
La∗∗∗32	7:55	Rest area	6	-45
Ca∗∗∗34	12:32	Learning area	2	-65
Ca∗∗∗lw	15:55	Learning area	4	-25
2d∗∗∗56	20:15	Learning area	8	-46

**Table 2:** Comparison of random models.

Model	Accuracy	Precision	Recall	*F*-measure
Random forest	59.93	61.14	59.47	59.95
GBDT	60.54	62.36	59.62	59.13
Xgboost	60.98	60.78	60.54	61.12

## Data Availability

The data used to support the findings of this study are available from the corresponding author upon request.
